# Using a Hybrid Multiattribute Decision-Making Model for Evaluating the Sustainable Development Potential of Characteristic Towns and Exploring Development Planning Strategies

**DOI:** 10.1155/2023/9065729

**Published:** 2023-01-31

**Authors:** Jing-Yang Lin, Lai-Chun Zhao, Yu-Yi Zheng, Qing-Kun Du, Lei Xiong, Bo-Wei Zhu, Gwo-Hshiung Tzeng

**Affiliations:** ^1^School of Art and Design, Guangdong University of Finance and Economics, Guangzhou 510320, China; ^2^School of Architecture and Allied Art, Guangzhou Academy of Fine Arts, Guangzhou 511400, China; ^3^Academy of Fine Arts, South China Normal University, Guangzhou 510631, China; ^4^Faculty of Humanities and Arts, Macau University of Science and Technology, Macau 999078, China; ^5^Graduate Institute of Urban Planning, College of Public Affairs, National Taipei University, 151, University Rd., San Shia District, New Taipei City 23741, Taiwan

## Abstract

In recent years, with the development of 'China's new urbanization, the “characteristic town movement” with the development of industrial economy first has brought problems to a large number of rural settlements, such as no cultural planning, no consumption of industry, and no soul. Then, in reality, there are still a large number of rural settlements under the planning of the upper-level local government, with the goal of developing into a characteristic town in the future. Therefore, this study believes that there is an urgent need to build a framework for evaluating the construction potential of rural settlements with sustainable characteristic towns. Not only that but also a decision analysis model should be provided for real-world empirical cases. This model needs to cover the assessment of the sustainable development potential of characteristic towns as the goal and the formulation of improvement strategies. This study combines the data collection of current characteristic town development rating reports, applies data exploration technology to extract core impact elements and obtain hierarchical decision rules, integrates expert domain knowledge with DEMATEL technology, and establishes an impact network relationship diagram between core impact elements. At the same time, the representative characteristic town cases are assessed for their sustainable development potential, and the modified VIKOR technique is applied to clarify the actual problems of the empirical cases, in an attempt to determine whether the development potential and development plan of the characteristic town meet the sustainable development needs from the pre-evaluation mechanism.

## 1. Introduction

One of the main global concerns in the shift from an agricultural rural society to an industrial modern society is urbanization. For instance, Goal 11 of the Sustainable Development Goals (SDGs) calls for making “cities and human settlements inclusive, safe, resilient, and sustainable” [1]. Future urbanization growth rates are anticipated to be primarily driven by India, China, and Nigeria, accounting for 35% of global growth from 2018 to 2050, even though the fact that developing countries are currently driving global urbanization, especially in Asia, Africa, and Latin America, which have large rural populations and are lagging. As an integral part of the urbanization process, the development of small towns is closely linked to rural areas [2–4]. Metropolitan areas prioritize the development of public infrastructure, health care, and education; villages with farming products, working populations, available open space, and cultural heritage are considered the hinterland for urban services; small towns in between act as the economic hinterland for large cities, providing primary employment, basic health, educational services, and public transportation for residents and nearby rural settlements [5–7]. Therefore, small towns can provide solutions for future urbanization and act as “network nodes” or rural “growth poles” [3, 5].

A hurdle for rural development in China has been the country's lagging infrastructure development. On the one hand, China's growing urban population has left the nation with housing shortages and environmental degradation [8]. On the other hand, China's rural development has been hampered by the country's slow infrastructure development. Premier Li Keqiang contends that creating characteristic towns to address the issues brought on by rapid urbanization is not only the route to economic success but also a vital strategy to reduce regional disparities given the current regional imbalance in China. As China's socio-economy transitions into a stage of transformation and innovative development, characteristic towns are a new type of industrial spatial organization. Characteristic towns are based on small platforms to achieve higher quality growth and demonstrate a way of developing local industries, preserving local cultural heritage, and establishing environmentally friendly urban life, generating a unique combination of local characteristics and endogenous institutions and systems oriented to create more socio-economic value [9]. It aims to improve urban and rural development patterns, promote economic transformation and upgrading, and promote new urbanization and rural revitalization. According to the National Development and Reform Commission's “Guidelines for the Standardized and Healthy Development of National Characteristic Towns,” all relevant departments in each region should coalesce to support the standardized and healthy development of characteristic towns around the five major aspects of grasping development positioning, planning the spatial layout, ensuring quality and efficiency, coordinating management mechanisms, and strengthening bottom-line constraints to further amplify the overall effect of the reform, while at the same time vigorously promoting industrial innovation and industrial upgrading with innovation as the base point, coordinating economic development and environmental protection, and promoting healthy and sustainable economic development in China.

Over time, China's characteristic towns have been vital in driving rural development in the following three ways, in addition to being a crucial component of the urban system: In order to promote the economic development of the rural population, characteristic towns first develop industrial systems based on the discovery of regional characteristics. Then, they use various methods to increase employment opportunities. Finally, through industrial development, economic upgrading, and transformation, they redesign the town's physical layout to be in harmony with the surrounding ecological environment and provide a suitable long-term living environment for a rural population [10]. Thus, it can be seen that different types of models have been established to promote economic development in China's characteristic towns and have undergone three stages of development processes, namely, long-term slow growth in the context of a planned economy (1949–1983), rapid development driven by township enterprises (1984–2002), and quality-oriented and differentiated development (2003–present) to continuously improve urbanization [11]. However, while developing rapidly, characteristic towns focus too much on regional/neighboring industries and face nonsustainable problems such as waste of resources, environmental pollution, and inefficiency [1]. On the one hand, China's rapid urbanization has led to a significant siphoning effect on large cities and the inevitable shrinkage of many satellite towns. At the same time, the aging of the population is more prevalent and growing in China. Therefore, the abovementioned issues will bring new challenges as well as add more complex difficulties to the construction of the present-day characteristic town projects. On the other hand, since the promulgation of the national white paper document related to characteristic towns, “several measures to promote the standardized and healthy development of characteristic towns,” national policies, and development plans, still to a great extent, widely promote the construction of characteristic towns as an important breakthrough in promoting new urbanization and the integration of urban and rural development. Therefore, the reality of the situation is that there are many areas of small-town construction that are scrambling, and even some towns do not pretend to learn from the successful model of the previous characteristic town construction projects to promote the development of the characteristic town. It is not difficult to infer that these projects are detached from their environmental conditions and cultural background and lack a long-term development plan, focusing more on short-term construction results. Thus, in the context of rural savvy shrinkage, how should the development potential of a characteristic town be explored and a sustainable development strategy is formulated based on the potential assessment is a matter of concern. This can help local governments to formulate long-term development plans for their characteristic towns in a more resource-efficient and realistic manner and to maximize the benefits of construction in the context of smart shrinkage to promote the sustainable development of their characteristic town projects in a continuous and phased manner.

To sum up, the purpose of this study is to evaluate the potential and development direction of the countryside to be developed in terms of its current situation and characteristics and to avoid the waste of resources caused by blind construction in the context of moving toward smart contraction. The subpurposes of this study contain the following three: (1) to extract the key elements of the construction planning of the characteristic town by reviewing the relevant literature and to construct a preliminary framework of assessment indicators for the sustainable development of the characteristic town; (2) to clarify the knowledge of the laws related between the core influencing elements and the development stages and ratings of the characteristic towns in the context of smart contraction; and (3) to analyze the performance of the representative existing characteristic town cases, evaluate the performance at the level of judging the development potential, and explore the sustainable and systematic design strategies for the real cases. To achieve the abovementioned research objectives, this study combines data collection of current characteristic town development rating reports and applies data exploration techniques to extract the core impact factors in the assessment framework. Also, we get the hierarchical decision rules, i.e., If…Then... Based on this, the DEMATEL technique is applied to integrate expert domain knowledge and establish the influence network relationship diagram between core influence elements. Finally, based on the results of the abovementioned study, an ex-ante assessment mechanism is constructed to determine whether the development potential and development plan of the characteristic town meet the sustainable development needs from a government-led perspective by applying the modified VIKOR technique to clarify the actual problems of the empirical cases, integrating the knowledge of hierarchical decision laws and the interfactor influence network relationships, and identifying the sources of influence behind the real problems.

## 2. Literature Review

Urbanization usually refers to the process of population concentration in cities, which leads to the expansion of cities and consequently causes a series of spatial, economic, and social structural changes. Currently, global urbanization continues to accelerate and is expected to rise from the current 56.2% to 60.4% between 2020 and 2030 according to the “World Cities Report 2020.” In the process of urbanization, western countries try to solve the problem of unbalanced development between large cities and rural areas, thus proposing the development model of small towns, and some cities have gradually evolved into a kind of industry-based “characteristic town”. For example, Provence in France, Greenwich in the United States, and Davos in Switzerland, with their long-standing regional culture, well-preserved ecosystems, and unique advantageous industries and education systems form the upgrading and transformation of the characteristic towns, guiding the optimization of the construction of Chinese characteristic towns [12]. China, facing the impact of urbanization, has likewise chosen the development model of small towns as a new form of industrial spatial organization as the socio-economy enters a phase of transformative and innovative development, to improve the urban-rural development pattern, to promote economic transformation and upgrading, and to promote new urbanization and rural revitalization. With innovation as the base, we will vigorously promote industrial innovation and industrial upgrading, coordinate economic development and environmental protection, and promote the healthy and sustainable development of China's economy.

The theory of “smart shrinkage” originates from the former socialism in eastern Germany, which proposed the management model of “fewer plans, fewer people, fewer buildings, and less land use” for cities. To date, the core idea of “smart shrinkage” aims to focus on sustainability, potential development dynamics, and reasonable city size while the city shrinks. Over time, scholars have observed that vacant villages in China have been widely reported, noting that a large number of townships are facing inevitable contraction at both the township and city levels [13]. This also confirms the development context and trends of the urban and rural environment in which a large number of Chinese characteristic towns are located. The concept of town construction faces these constraints and challenges from the general environment, and it should not be overlooked that the level of development of characteristic town projects is significantly influenced by the scale of the local urban and rural economic and social structures. At present, on the one hand, the country promulgates the white paper document related to the characteristic town, “promoting several measures for standardized and healthy development of characteristic town,” which still greatly and widely promotes the construction of characteristic town as an important breakthrough to promote the new urbanization and the integration of urban and rural development. Therefore, the reality of the situation is that there are many regions, especially in the northeast, southwest, and other remote areas of the town construction that is scrambling, and even some towns do not pretend to learn from the successful model of the previous characteristic town construction projects to promote the development of the characteristic town. On the other hand, it is not difficult to find that it is still difficult to reverse the demographic problems faced by urban and rural areas while promoting the construction of characteristic towns based on real-life cases. For example, the town of Sunshine in Changzhou, Jiangsu Province [14], the “red culture town” of Nanniwan in Yan'an, Shaanxi Province [15], and the “cultural and sports” town of Kangping, Shenyang, Liaoning Province [16] have been built, but they are still shrinking without relief. According to relevant data from the National Bureau of Statistics, the aging population in Changzhou City, Jiangsu Province surged from 449,000 (9.8%) in 2010 to 1,056,000 (20.01%) in 2021; areas such as Shaanxi Province and Liaoning Province also show a rising trend of about 7% population aging. For instance, Yan'an City in Shaanxi Province experienced a rural population loss of about 247,000 from 1,129,000 to 882,000 between 2010 and 2021, and other areas mentioned above also experienced different degrees of population decline. Therefore, there are sufficient reasons to infer that the old construction strategy and project management thinking of the characteristic town can hardly achieve the expected construction goals and benefits in the context of gradual urban and rural contraction.

In the characteristic town construction project, the satisfaction of local people, the coordination of government departments, the rationality of town planning, and the selectivity of core industries all have a significant impact on the decision. To ensure the development of characteristic towns towards high quality, relevant scholars have analyzed the existing town cases with different assessment methods. This includes selecting the integrated MCDM method, constructing a development strategy map for urban and rural tourism/town tourism using four aspects (cultural preservation, environmental support, economic development, social awareness) with the DEMATEL method, establishing component scores in each aspect of the principal component analysis (PCA) method, and then evaluating the weights of each aspect/component using the analytical network process (ANP) method to evaluate the competitive advantage of urban and rural tourism using VIKOR [17]. By collecting, screening, and rationally analyzing comprehensive evaluation indexes, we constructed a comprehensive evaluation index system for the development of agricultural characteristic towns from five aspects, including economic development, social progress, ecological environment, urban-rural integration, and modern agriculture and conducted an empirical study on the development status of 13 national first and second batch agricultural characteristic towns in three northeastern provinces using the TOPSIS method [18]. It is not difficult to find that previous studies have focused on the postevaluation of completed characteristic town projects, with little consideration of ex-ante evaluation and a lack of consideration in the context of promoting urban and rural areas toward smart contraction.

## 3. Methods and Steps

The research methods and technical lines applied in the different phases of this study and the corresponding research questions addressed are shown in Figure 1. The methodological model applied in this study is considered as a hybrid multiattribute decision model, consisting of three analytical techniques. First, the rough set theory (RST) was proposed by Polish scholar Pawlak in 1982, and the method has been developed and widely used in the fields of machine learning, knowledge acquisition, and decision analysis. The rough set theory considers knowledge as the ability to classify real or abstract objects. RST can be used to handle quantitative and qualitative attributes simultaneously without requiring a priori information regarding the probability distribution of the data. Many studies have adopted the RST approach to extract rules and patterns from collected data or unclassified information, such as analyzing urban watersheds morphometrics in arid and semiarid regions [19], tourism marketing analysis [20], and energy consumption in buildings [21].

Secondly, the second analytical technique in the decision model is the decision laboratory analysis-based network analysis (DANP) method. DANP technique used the basic concept of the ANP technique by applying the influence matrix of the DEMATEL technique. In evaluation studies, the application of this method permits the existence of interinfluence relationships among the criteria in the evaluation framework and clarifies the influence of network relationships (INRM) between the evaluation constructs and the criteria. On the other hand, compared to the traditional ANP technique, the DANP technique overcomes the unrealistic assumption of equally important influence roles among the constructs in the assessment framework. The influence degrees among dimensions are used to weight the unweighted supermatrix, which leads to a weighted supermatrix. Finally, in the empirical research phase, the DANP technique is followed by the application of the modified VIKOR (mV) technique, which improves on the traditional VIKOR method by setting the best and worst values, replacing the best performance value among several scenarios with the desired level [22]. In recent years, the DANP-mV model has been widely applied in the field of urban design and regional development planning, and Zhu et al. [23] applied the DANP-mV model to explore the improvement strategies of urban public open spaces to move towards a healthy aging society. Zhang et al. [24] applied the FDM-DANP-mV model in conjunction with fuzzy theory to explore sustainable development plans for catch-up universities. The same multiattribute decision model was also used to explore age-friendly improvement strategies for urban neighborhood green spaces under public health orientation [25].

### 3.1. Rough Set Theory (RST)

Rough set theory (RST) is an analytical method used to solve the imprecise knowledge relationship between conditional attributes and decision-making attributes in classification functions [26]. The specific steps are described as follows:

 
*Step 1.* We build the information system. An information system *S* = (*U*, *A*), where *U* and *A* are nonempty finite sets is called the universe of objects *U* and the set of attributes *A*.
 
*Step 2.* We confirm the undistinguishable relation. For any subset of conditional attributes *B* ⊂ *C*, the relevant equivalence relations can be defined as IND(*B*) = {(*x*, *y*) ∈ *U*|∀*a* ∈ *B*, *f*_*a*_(*x*) = *f*_*a*_(*y*)}.
 
*Step 3.* The upper and lower bounds are set. *I*_*B*_[*x*] is the equivalence class function of the subset of attributes *B* for each object. Get the lower approximation set $\underline{B}X$ and the upper approximation set $\bar{B}X$. The difference between these two sets is what we consider the boundary region of the decision domain. The boundary region is used to describe the classification quality of the dataset.
 
*Step 4.* We confirm the dependency of the conditional attributes. The full domain *U* is partitioned by the indistinguishability relation of the decision attribute D as *U*/IND(*D*) = {*D*_1_, *D*_2_,…, *D*_*k*_}. In the formula *U* = ∪_*i*∈{1, ⋯,*k*}_*D*_*i*_, *BD*_*i*_ is the lower approximation bound of each subset of the conditional attribute *B* for the decision attribute D. It also represents the positive domain range of the decision attribute, from which POS_*B*_(*D*) is derived.
 
*Step 5.* We derive behavioral law knowledge. The approximation of the set of conditional attributes will maintain the correlation between conditional attributes and decision levels. Therefore, for decision analysis, a set of decision rules can be derived from the decision table, such as the decision rule in *S* denoted as Φ⟶Ψ and read as ifΦ, thenΨ.

### 3.2. Decision Analysis Laboratory-Based Network Analysis (DANP)

More and more scholars in the field of operations research have been trying to introduce the Decision Analysis Laboratory (DEMATEL) method into multicriteria decision models and to train the weights of evaluation indicators by combining the basic concepts of network analysis (ANP), which allows for the interaction between evaluation indicators. The specific calculation steps of the DANP technique are described as follows:

 
*Step 1.* We establish the direct influence relationship matrix *Z*. The data were collected from the expert questionnaire, and the scale scores in the questionnaire include 0, 1, 2, 3, and 4, where 0 represents the semantic meaning of no influence and 4 means highly influential.
 
*Step 2.* We establish the average direct impact relationship matrix *P*.
 
*Step 3.* We conduct the consensus test of the expert questionnaire. The consensus level of the expert questionnaire is checked by calculating the average gap ratio.
 
*Step 4.* We build the regularized average direct impact relationship matrix *M*.
 
*Step 5.* We build the total influence matrix *T*. As the power of the matrix *M* tends to infinity, the indirect influence contained in this matrix will continue to decrease, so it is necessary to build an inverse matrix of the difference between the unit matrix *I* of *n* × *n* and the matrix *M*. The total influence matrix *T* can be obtained by matrix multiplication of this inverse matrix with the matrix *M*
 
*Step 6.* We plot the INRM.
 
*Step 7.* We create the unweighted supermatrix *W*^*α*^.
 
*Step 8.* We build and calculate the limiting weighted supermatrix *W*^*g*^.

### 3.3. Modified Compromise Sorting Method (mV)

The modified VIKOR technique improves the setting of positive-ideal solutions and negative-ideal solutions in the traditional VIKOR technique. The specific calculation steps are as follows:

 
*Step 1.* We compensate for the shortcomings of the traditional VIKOR method. We set the aspiration level and the worst value as the positive and negative-ideal solutions for each indicator, respectively.
  Desire level *f*^aspire d^=(*f*_1_^aspire d^ ⋯ , *f*_*j*_^aspire d^, ⋯, *f*_*n*_^aspire d^), where *f*_*j*_^aspire d^ represents the level of desire, or what is called the optimum value.
  Worst value *f*^worst^=(*f*_1_^worst^, ⋯, *f*_*j*_^worst^, ⋯, *f*_*n*_^worst^), where *f*_*j*_^worst^ represents the worst value.
  In this subject, the rating scale in the performance evaluation questionnaire is from 0 to 10 (very poor←0, 1, 2,…, 9, 10 ⟶ excellent). Therefore, a score of 10 can be considered as reaching the desired level, and a score of 0 is the worst value. Therefore, *f*_*j*_^aspire d^=10 is the level of desire. *f*_*j*_^worst^=0 is the worst value.
 
*Step 2.* We define the gap value. First, we need to calculate the difference between the aspiration level and the performance score of the case to be rehabilitated on each evaluation index, *J*, and the difference between the aspiration level and the worst value, *K*. We obtain the gap values of the case to be rehabilitated on each evaluation index by the product of the ratio of the two and the corresponding index impact weights (IWs).

## 4. Results and Discussion

### 4.1. Data Exploration Analysis of Characteristic Town Cases

The research collects case data on characteristic towns in mainland China. Considering the differences in regional economic development and population size and urbanization development process, this study mainly investigated 178 case studies of characteristic towns in Zhejiang Province and Guangdong Province, China. At the same time, by reviewing previous studies, this study summarizes 16 environmental factors that are closely related to the sustainable development potential of the characteristic towns (Table 1). Most of the characteristic towns are related to tourism and leisure [12], so these 16 environmental elements were mainly selected from an evaluation system based on sustainable development of urban and rural tourism. This study is very similar to the direction of the assessment of characteristic towns towards sustainable development explored in this paper, and both emphasize rethinking the balance and harmony of local society, environment, and regional economy by applying a modern perspective of regional and sustainable development [17]. Besides, this study also looks for elements related to other development studies of characteristic towns. On the one hand, the sustainable development path of the characteristic town is proposed to a great extent from the perspective of environmental support and cultural preservation based on the advantages of local natural resources and location. On the other hand, its sustainable development path is studied from the social consciousness level of urban-rural identity and urban-rural communication [34].

These 16 environmental factors are considered conditional attributes, and the official public ratings of the current development of 178 characteristic towns are considered decision attributes. The study then invited experts from the Zhejiang and Guangdong provinces of China to form focus groups, and a total of 17 experts were invited to multiple rounds of meetings. These experts were mainly from the fields of the regional economy, local policy, and urban planning. Each expert was required to have a master's degree or higher and more than 10 years of work experience, and all had been involved in the practice and research of China's characteristic town construction projects. After several rounds of meetings, the interviewed experts were asked to classify 178 characteristic towns by 16 environmental factors (as shown in Table 2) to obtain data on the conditional attributes.

Data exploration techniques are used to obtain core condition attributes and build knowledge of hierarchical decision laws (i.e., If...Then...rule). As shown in Table 3, the classification quality of the data collected in this study is 0.966, and the classification accuracy of each rank is 0.684, 1.000, 0.937, and 1.000, respectively, which indicates that the data have a certain degree of roughness and high classification accuracy.

The importance of each conditional attribute can be obtained by RST calculation based on its dependence at different levels. Three of the 16 conditional attributes were found to have a high degree of importance and were therefore classified as core conditional attributes (Table 4). In addition, RST provided 22 rank decision rules, among which there were 2 ***D*** = 1 rules, 6 ***D*** = 2 rules, 10 ***D*** = 3 rules, and 4 ***D*** = 4 rules. In this study, the rules covering more than 10% were extracted one by one, as shown in Table 4.

Four of these six rules reveal that the main environmental conditions for a characteristic town project to be rated as “best” by local policymakers are stable and effective local policies, a vibrant urban and rural economy, and an excellent living environment with well-developed infrastructure services. In terms of socio-cultural assets, it is important to pay attention to and preserve historical sites such as industrial heritage buildings in the area and to promote the residents' sense of identity with the local culture. The analysis shows that the creation of natural landscape and living environment is related to the establishment of the local identity of residents, which is also the basis for promoting urban-rural communication. As Ziyaee [35] points out, the physical environment characteristics of urban and rural areas are only one aspect of improving the quality of urban and rural identity of residents; the influence of nonphysical environment aspects is also extremely significant. The nonphysical environment involves specific events and activities in public space that can shape public memory and public life in urban and rural areas, which form different levels of local identity. On the other hand, this study's interpretation of the data analysis is close to Sasaki's [36] finding that characteristic towns also need a “culture-based production system,” a balanced system of cultural production, and consumption that utilizes accumulated cultural capital. A so-called successful town project should be based on socially inclusive and grassroots empowerment.

Two rules in Table 4 explain how a town is judged to be in the “worst” state of development when it is characterized in various ways. This study concludes that the conditional attributes involved in rules 5 and 6 may be important factors that lead to the nonpermanent development of a town and that these factors are correlated with the positively influenced conditional attributes mentioned above. This study argues that before the construction of a characteristic town project, the site selection and policy evaluation stages should be examined to see whether the region has significant local cultural characteristics or architectural style and whether the town has the basis for tapping into the folk culture and developing festivals and events. At the same time, the local industry brand effect, development potential, and local employment should be evaluated. The fieldwork revealed that in Jiangsu, Zhejiang, and Guangdong, where the concept of township collectivity is strong, it is an honor to be called a “village squire” and there are many precedents of successful participation of village squires in the governance of villages and towns, and they have made immeasurable positive contributions to the funding base of public affairs, external communication, and resource integration. Not only in Jiangsu, Zhejiang, and Guangdong but also in China, there are a large number of small towns and villages that are formed by clans because of blood ties, and religion does not play a significant role in village governance. Therefore, the governance and transformation of the Chinese countryside have to be done within the network formed by the unique human, blood, and cultural traditions. As one can imagine, once this rural structure is destroyed and there is no other force to fill the gap, not only is the governance of the countryside impossible but also the original blood and cultural network will be destroyed, changing the existing rural landscape and cultural structure.

### 4.2. Performance Evaluation and Improvement Strategies for Empirical Cases

#### 4.2.1. Case Description

This study takes CuiHengCun (CHC) in Zhongshan City as an empirical case, where agriculture has long been the leading industry. The local government has paid attention to the development of the architectural heritage, supplemented by the ecological protection and management of the natural landscape of the village, while shaping the new cultural industry of the town around the celebrity effect tourism of “Sun Yat-sen's former residence.” The existing buildings in the village are mainly Qing Dynasty and Republican buildings, mostly in the style of western-style classicism popular at the end of the 19th century and the Lingnan architectural style houses built in the Qing Dynasty (about 90 houses). In addition, the historical and cultural resources promote the cultural value-added empowerment of the region. In addition to the former residence of Sun Yat-sen, the village also has the former residence of Yang Yin and the former residence of Lu Haodong, which are listed as provincial cultural heritage units in Guangdong Province. In addition to architectural culture, the CHC has a long history and culture, and the commercially developed former residences of historical celebrities and many natural and historical relics together form the unique tourism and cultural resources of this region. On the other hand, CHC holds a variety of folk cultural festivals every year. In addition, the village buildings require the application of traditional crafts such as wood carving and gray carving. Therefore, the village's tangible and intangible cultural heritage still exists and affects the daily life of local villagers and has been stably inherited.

The CHC is located in the southeast of Zhongshan City, east of the Pearl River mouth Lingding Ocean, the north and west are surrounded by hills with short elevation, the highest Yunti Mountain is 268 meters above sea level, and the famous natural scenery is Golden Penang Mountain, Yunti Mountain, Wugui Mountain, and other landscape areas. The superior geographical location adjacent to the sea port makes it easy for residents to go to the sea. Historically, the CHC has a large number of people who went abroad to make a living, and the return of overseas Chinese brought foreign architectural styles and craftsmanship to the CHC. Due to its geographical location, the CHC has generated a rich industrial chain that allows the residents to maintain their traditions and continue to practice agriculture (rice and mixed grains mainly). Secondly, the geographical factor of being near the sea allows the villagers to stay engaged in peri-sea farming and fishing. In addition to the original local primary industry, the regional government, in conjunction with developers, has also developed the tertiary industry around the theme of celebrity culture and historical culture, complementing the tourism resources within the Pearl River Delta.

#### 4.2.2. Influence Weights and Network Relationships among Conditional Attributes within Rules

In this study, the DEMATEL technique was applied to analyze the interinfluence network relationship between indicators, and the calculation results are shown in Figure 2. Among the indicators concerning the characteristic town with high sustainable development potential, the highest influence weights (IWs) are urban-rural identity (**SC**_1_) and economic activities (**ED**_2_). This suggests that, on the one hand, a high level of historical and cultural identity and regional environmental identity in the area are to be developed into a characteristic town, whether it is affiliated with local villagers or foreign tourists is conducive to the dissemination of local regional culture, while using cultural elements to stimulate innovation, revitalize traditional industries, and promote a more comprehensive industrial chain [37]. On the other hand, whether urban and rural economic activities are active or not is also an important potential factor as a characteristic town towards efficient development; if a unique local industrial activity can be supported and new business opportunities are created through a common sense of urban and rural residents, more diverse talents will be attracted to join the town and achieve industrial development. In addition, the core indicators of RST results also include economic activity (**ED**_2_), and this study suggests that the traditional industries and the surrounding industries to be developed should be evaluated as a whole before the construction of a characteristic town project, to explore the local industrial resources and establish its economic advantages.

Although the IWs are not high, the dominant source of influence is policy promotion (**SC**_4_). Therefore, this study suggests that in terms of economic factors, relevant policymakers should use “capital-based” overall planning for the development of characteristic towns and promote the integrated development of local socio-economic, environmental, and cultural aspects around characteristic towns [38]. At the level of noneconomic factors, future development proposals should be made from different perspectives of the overall planning of the characteristic town, such as ecological construction, history and culture, and characteristic industries [39]. At the same time, policy measures should be “tailored” to the local situation, problems, and context [9]. This suggests that policymakers should also propose strategies for the conservation and restoration of historic buildings and relics and that the spontaneous conservation of historic sites by local villagers should be achieved through the life experiences and aesthetic preferences of folk artisans, which will increase their economic income and enhance their sense of local identity, achievement, and affinity. The second is the historic sites (**CP**_2_). Secondly, as a secondary indicator, historical sites (**CP**_2_) should be maintained by both urban and rural residents. This will not only enhance the sense of identity of urban and rural residents with such historical elements but also attract foreign tourists to a certain extent and greatly promote the development of the local tourism industry.

In the interactive network relationship in Figure 3, the highest influence weight (IWs) is the urban-rural identity (***SC***_1_), which indicates that if the urban-rural identity of local culture and historical sites is low, on one hand, it leads to the inability to attract foreign talents to increase employment opportunities, which affects the industrial development within the town to a greater extent; on the other hand, it leads to the inability of the urban-rural residents to gather their strength to jointly maintain the local. On the other hand, the residents of urban and rural areas are not able to work together to maintain the existing historical sites, which affects the tourism development of the town. In the RST decision rule, even if there are a small number of job opportunities and some talents remain in the area, if it is found that the urban and rural residents' sense of identity and belonging to the area is extremely weak, and there is almost no natural landscape in the area to stop and enjoy, it is still decided that the characteristic town does not have any development potential. Second, the state of the physical environment within the town and countryside is also particularly important. If the region lacks buildings with significant local cultural characteristics or natural landscapes with great regional characteristics, it will not be able to attract foreign tourists and promote the development of the town's industry.

#### 4.2.3. Performance Evaluation of Empirical Cases and Suggestions for Improvement of Problems

Through the modified VIKOR method analysis, the deficiencies in the current situation of the empirical case (CHC) are highlighted in the perspective of the construction of the characteristic town. Although the overall development potential of the CHC seems to be high, it is easy to find that there is too much lack of spatial places that reflect the production and operation methods of the village. In addition, the evaluation data (Table 5) show that the residents have a low sense of cultural identity and a relative lack of economic activities in the village and the surrounding area. The current strength of the village is its ability to provide a higher quality of living environment to both residents and outsiders. The results of the performance assessment reveal that although the CHC is strategically located and has a rich industrial chain, there is still a lack of resources such as industrial relics with some historical and cultural value. In the long run, this will further exacerbate the lack of urban and rural identity of the local people and make it difficult to maintain a sufficient labor force and promote the incubation of cultural/creative industries. In addition, this study also found that top-down policy support, publicity, and promotion in CHC are not strong and accurate enough. The local government should pay attention to the construction of business culture in this village and town and further strengthen the guidance and promotion of policy and culture.

According to the relevant information, the CHC has long been dominated by agriculture, but in recent years, it has made efforts to develop the cultural tourism industry around the historical and cultural heritage such as “Sun Yat-sen's former residence.” There is a lack of material spatial carriers that can reflect local traditional industries, characteristics, and history in the current situation of the village. Compared with historical celebrities, local characteristic industries that are closer to the daily lives of residents can better reflect collective memory and gain a wider sense of identity. Therefore, this study suggests that cultural elements and symbols with characteristics of farming civilization, regional features, and national characteristics should be integrated into related industries such as agricultural products processing and manufacturing, agricultural tourism, and farming experience, giving more cultural significance to these industries, promoting the transformation and upgrading of village landscape and rural architectural space with innovative thinking, and promoting the construction of characteristic towns and the integrated development of rural cultural tourism.

In addition, it is of the concerns that the current sense of local identity among the local population of the CHC is low. Previous research has long suggested that community tourism developed around cultural heritage needs to create a strong and stable sense of place and identity [40]. The construction of a sense of local identity is related to the attractiveness and branding of a characteristic town [41], and the lack of identity of the local population exacerbates the difficulty of developing the necessary human and labor resources needed to develop a characteristic town in CHC, a village with an already small and aging population. In the data exploration stage of this study, Table 4 also suggests that when the local industry remains are well preserved and can present the traditional production and historical characteristics of local life intact and when residents generally have a strong sense of local cultural identity, the village has the potential to develop into a sustainable town with characteristics. Therefore, this study suggests that local governments should actively promote traditional industries or local industries with characteristics to improve the economic situation of the industries and deepen the sense of local identity and local connection. In the past, if the production-based traditional industries wanted to transform to make use of cultural value-added, they needed to make a breakthrough in the concept first, from focusing on manufacturing products to focusing on consumers' feelings, evolving from material production to knowledge economy, experience economy, and aesthetic economy. The “creative life industry” in Taiwan's cultural and creative industries is a classification different from other foreign cultural industries, which integrates the core knowledge of life industry with creativity and is an industry that provides high-quality aesthetics and deep experience, echoing Taiwan's trend toward sophistication, creativity, and high quality.

Based on the understanding of the development of characteristic towns in mainland China in the past decade, this study concludes that the government should not emphasize hardware facilities in the process of promoting small town projects; for areas where the urban economy is not yet developed, the government should not rely too much on small towns to achieve the purpose of economic development but should first focus on the advantageous resources to develop the urban economy; the construction of characteristic towns should be tailored to local conditions and should not copy the experiences and models of other places; characteristic towns can be promoted in all aspects and take the diversified and market-oriented route as much as possible. The results of this study, in Figure 2, also show the dominant influence of policy promotion in endowing characteristic town projects with perpetual development potential. It can significantly influence important local development influences such as the governance of the local landscape, the clustering and support of industries, and the customization of the supporting welfare system. On the other hand, the results of this study also suggest that the current strength of the village lies in its ability to provide a good living environment to both residents and foreign visitors. Zou and Zhao [42] have emphasized the need for characteristic towns to emphasize small-scale and beautiful planning and livable environments as a source of creative inspiration for attracting innovation and talent. Many local governments and project campers have realized that cultural and art creative workers and investors have a high demand for a quality living environment and they are highly mobile. This study suggests that CHC villages should take a step up in eco-environmental protection concerning existing real-life cases, for example, the planning of characteristic towns requires planning according to the standard of scenic spots of grade 3*A* or above. This requirement does not require all characteristic towns to assume tourism functions, but it does require them to create a better environment to attract and retain residents.

## 5. Conclusion

By summarizing the relevant literature, this study initially constructs a framework for assessing the sustainable development potential of characteristic towns before construction. This framework is useful for assessing the existing local cultural resources before the construction of a characteristic town project to avoid the waste of resources by blindly implementing relevant policies. Then, by analyzing data from 178 completed cases of Chinese characteristic towns, this study identifies three core condition attributes that influence the formation of the sustainable development potential of characteristic towns. It also clarifies the regular knowledge of the environmental characteristics of rural settlements and their potential for sustainable development of characteristic towns (i.e., If...Then...rule). In traditional assessment studies, the extraction of assessment criteria and the diagnosis of current problems rely more on expert empirical knowledge. In contrast, this study attaches importance to clarifying the core condition attributes from objective data of real cases and developing the relevant regular knowledge between the environmental conditions of villages and the potential for sustainable development of characteristic towns.

RST-DANP-mV was developed and applied in this study to achieve the integration of the relevant law knowledge embedded in real cases and expert domain knowledge in the evaluation analysis of empirical cases. This study further analyzes the key intercriteria that influence network relationships and influence weights. Then, the local environmental conditions of the CHC are assessed, and the deficiencies and problems in the current environmental conditions of CHC are identified through the modified VIKOR technique. Following a dual knowledge-driven decision path, this study aims to discover the sources of influence behind real-world problems and provide systematic suggestions for improvement in the development of CHC's characteristic town development potential.

The limitation of this research is that based on the feasibility of the case study of characteristic towns, all realistic cases in the data exploration phase of this study are from the characteristic towns that have been built in China in the past 30 years. On the other hand, in this study, the rating data on the development status of the completed characteristic town cases are mainly based on the evaluation reports of the characteristic town construction projects by the government departments that are publicly available. Therefore, there are assumptions about the credibility of the government's publicly available project evaluation reports in this study. In addition, the recommendations for enhancing the development potential of the characteristic town developed in this study are only for the empirical case (CHC) and are not suitable to be provided to other villages that have the development vision of building into a characteristic town. However, the decision analysis model constructed in this study and the idea of potential enhancement strategy development can be applied to other relevant cases. This study concludes that in the future, a large number of empirical cases from the same region can be evaluated for the current situation, and a nonadditive approach-fuzzy integral can be used to complete the evaluation and ranking of the potential of multiple village cases for the perpetual development of a characteristic town.

## Figures and Tables

**Figure 1:** Model procedure for new multiple criteria decision making for creating the best sustainable improvement strategies.

**Figure 2:** The INRM (influential network relation map) of total influence relationships (*D* = 4).

**Figure 3:** The INRM (influential network relation map) of total influence relationships (***D*** = 1).

**Table 1:** Primary evaluation framework.

Dimensions/attributes	Descriptions	Cited references
*Cultural preservation (CP)*		
Settlement landscape (***CP***_1_)	Preserving the unique settlement and common features through the awareness of urban and rural residents.	[17, 27]
Historical sites (***CP***_2_)	Preserving the local culture and historical monuments through the awareness of urban and rural residents.	[17, 28]
Festivals & ceremonies (***CP***_3_)	Continuously promoting the local folk festivals and religious celebrations through awareness of urban and rural residents.	[17, 29]
Traditional arts activities (***CP***_4_)	Inheriting local folk skills and arts and promoting traditional folk-art activities through awareness of urban and rural residents.	[17, 29]

*Environment sustentation (ES)*		
Geographical landscape (***ES***_1_)	Maintaining the unique local geographic and geologic landscape through the common power of urban and rural residents.	[17, 27]
Industrial relic (***ES***_2_)	Maintaining the unique industry relics and promoting local industrial activities through the common power of residents.	[17, 28, 30]
Living environment (***ES***_3_)	Maintaining and improving the local living environment quality through the awareness of urban and rural residents.	[17, 31]
Leisure & recreation field (***ES***_4_)	Maintaining and improving the service quality of local leisure and recreation fifields through the awareness of urban and rural residents.	[17, 32]

*Economic development (ED)*		
City & countryside empowerment (***ED***_1_)	Promoting city and countryside empowerments and nurturing a unique local industry through the common consciousness of urban and rural residents.	[12, 17, 32, 33]
Economic activities (***ED***_2_)	Promoting unique local industrial activities and creating new business opportunities through the common consciousness of urban and rural residents.	[12, 17, 31, 33]
Investment incentives (***ED***_3_)	Attracting foreign investment and resources to aid urban and rural development through local business and economic activities.	[17, 32, 33]
Employment opportunities (***ED***_4_)	Promoting local employment opportunities and attracting talents to return home through local business and economic activities.	[17, 31, 33]

*Social consciousness (SC)*		
Urban and rural identification (***SC***_1_)	Promoting the sense of identity that urban and rural residents feel toward local culture and historical sites.	[17, 34]
Urban and rural exchanges (***SC***_2_)	Enhancing the urban and rural competitiveness by learning and exchange among different urban and rural residents.	[17, 34]
Industrial common prosperity (***SC***_3_)	Maintaining the prosperity of urban and rural industries by residents' businesses and visitors' concerted efforts.	[12, 17]
Policy promotion (***SC***_4_)	Creating rural and urban features and developing rural and urban economic activities through urban and rural policy promotion.	[12, 17, 32]

**Table 2:** Conditional attributes and semantic scale.

Dimensions	Attributes	Semantic scale
Cultural preservation (*CP*)	Settlement landscape (***CP***_1_)	1 = almost none, very scarce
		2 = with 1–2 settlements
		3 = more surviving settlements
		4 = almost always for settlements
	Historical sites (***CP***_2_)	1 = almost none, very scarce
		2 = with 1–2 historical sites, lack of protection
		3 = with some ruins and a variety of historical and cultural monuments, basically preserved
		4 = historical sites and a variety of historical and cultural monuments are well preserved throughout the area
	Festivals & ceremonies (***CP***_3_)	1 = almost none, very scarce
		2 = with 1–2 traditional festival ceremonies with less resident participation
		3 = several holiday ceremonies each year, with most residents participating
		4 = very frequent, large scale, with regional influence
	Traditional arts activities (***CP***_4_)	1 = almost none, very scarce
		2 = with 1–2 traditional art activities, less residents participate
		3 = several traditional art activities, most residents participate
		4 = very frequent, large scale, with regional influence
Environment sustentation (*ES*)	Geographical landscape (***ES***_1_)	1 = almost none, very scarce
		2 = a few natural landscapes
		3 = some existing natural landscapes
		4 = adequate and high-quality natural landscape
	Industrial relic (***ES***_2_)	1 = almost none, very scarce
		2 = a few industrial sites
		3 = some of the surviving industrial sites
		4 = industrial sites throughout
	Living environment (***ES***_3_)	1 = poor living environment and low recognition by residents/visitors
		2 = average living environment and multiple improvement needs still exist
		3 = well-living environment to meet basic living needs
		4 = excellent living environment with excellent supporting facilities
	Leisure & recreation field (***ES***_4_)	1 = almost none, very scarce
		2 = a few recreational facilities are available
		3 = some existing recreational facilities
		4 = recreational facilities throughout
Economic development (*ED*)	City & countryside empowerment (***ED***_1_)	1 = weak awareness of urban and rural residents and lack of cultivation of local specialty industries
		2 = general awareness of urban and rural residents, with a few local specialty industries
		3 = good awareness of urban and rural residents and some local special industries exist
		4 = better awareness of urban and rural residents spread across local specialty industries
	Economic activities (***ED***_2_)	1 = urban and rural residents have no intention to participate, and there is a great lack of business opportunities for industrial innovation
		2 = low participation of urban and rural residents and few industrial innovation business opportunities
		3 = urban and rural residents choose to participate in some existing industry innovation business opportunities
		4 = basic participation of urban and rural residents and innovative business opportunities throughout the industry
	Investment incentives (***ED***_3_)	1 = foreign investment resources are very scarce and urban and rural development is slow
		2 = few foreign investment resources and average urban and rural development
		3 = some foreign investment resources available and good urban and rural development
		4 = large amount of foreign investment resources and faster urban and rural development
	Employment opportunities (***ED***_4_)	1 = employment opportunities are very scarce and talent attraction is lacking
		2 = few job opportunities, attracting few talents
		3 = have some employment opportunities and attract some talents
		4 = large number of job opportunities, attracting large number of talents
Social consciousness (SC)	Urban and rural identification (***SC***_1_)	1 = low identification with local culture and history among urban and rural residents
		2 = urban and rural residents generally identify with local culture and history
		3 = urban and rural residents identify well with local culture and history
		4 = urban and rural residents have a high degree of identification with local culture and history
	Urban and rural exchanges (***SC***_2_)	1 = lack of communication between different residents in urban and rural areas and low competitiveness of urban and rural areas
		2 = general exchange between different residents in urban and rural areas and general competitiveness in urban and rural areas
		3 = general exchange between different residents in urban and rural areas and good competitiveness between urban and rural areas
		4 = frequent exchanges between different residents in urban and rural areas and outstanding urban-rural competitiveness
	Industrial common prosperity (***SC***_3_)	1 = lack of cooperation between residents (businesses) and tourists and lack of urban and rural industries
		2 = small amount of cooperation between residents (businesses) and visitors and urban and rural industries in general
		3 = residents (businesses) and tourists cooperate commonly and good urban and rural industries
		4 = frequent cooperation between residents (businesses) and tourists and prosperous industries in urban and rural areas
	Policy promotion (***SC***_4_)	1 = lack of urban and rural policy promotion and slow development of urban and rural economic activities
		2 = general promotion of urban and rural policies and general development of urban and rural economic activities
		3 = the promotion of urban and rural policies is widespread, and economic activities in urban and rural areas are developing well
		4 = high intensity of urban and rural policy promotion and good development of urban and rural economic activities

**Table 3:** Quality approximation of decision classes.

Class no.	Of objects	Lower approximation	Upper approximation	Accuracy
1	15	13	19	0.684
2	32	32	32	1.000
3	93	89	95	0.937
4	38	38	38	1.000
Quality of classification		0.966		

**Table 4:** Minimal covering rules with strength exceeding 10% in decision = 4/1.

Core attributes	Living environment (*ES*_3_), economic activities (*ED*_2_), urban and rural exchanges (*SC*_2_)	
Rule no.	Core level decision rules	
1	***ES***_3_ = 4, ***SC***_4_ = 4	Good class (***D*** = 4) (76.32%)
2	***ES***_2_ = 4, ***SC***_1_ = 4	Good class (***D*** = 4) (18.42%)
3	***ED***_2_ = 4, ***SC***_4_ = 3	Good class (***D*** = 4) (15.79%)
4	***CP***_2_ = 4, ***ES***_2_ = 4	Good class (***D*** = 4) (10.53%)
5	***CP***_1_ = 1, ***CP***_4_ = 1, ***ED***_1_ = 1	Poor class (***D*** = 1) (66.67%)
6	***ES***_1_ = 1, ***ED***_4_ = 2, ***SC***_1_ = 1	Poor class (***D*** = 1) (26.67%)

**Table 5:** Assessment results of the current situation of the CHC in terms of moving towards the construction of a characteristic town.

Criteria	Influence weights (IWs)	CuiHengCun (CHC)
		Gap ratio
Urban and rural identification (***SC***_1_)	0.207	0.375
Policy promotion (***SC***_4_)	0.111	0.375
Industrial relic (***ES***_2_)	0.126	0.463
Living environment (***ES***_3_)	0.188	0.300
Economic activities (***ED***_2_)	0.197	0.375
Historical sites (***CP***_2_)	0.171	0.363

## Data Availability

The data used to support the findings of this study are included in the article.
